# Comparing Machine Learning Methods to Improve Fall Risk Detection in Elderly with Osteoporosis from Balance Data

**DOI:** 10.1155/2021/8697805

**Published:** 2021-09-09

**Authors:** German Cuaya-Simbro, Alberto-I. Perez-Sanpablo, Eduardo-F. Morales, Ivett Quiñones Uriostegui, Lidia Nuñez-Carrera

**Affiliations:** ^1^Instituto Tecnológico Superior del Oriente del Estado de Hidalgo (ITESA), Carretera Apan-Tepeapulco Km 3.5, Colonia Las Peñitas, Apan Hidalgo, Mexico; ^2^Instituto Nacional De Rehabilitación Luis Guillermo Ibarra Ibarra (INR-LGII), Mexico-Xochimilco Av. 289, Arenal de Guadalupe, 14389 México City, Mexico; ^3^Instituto Nacional de Astrofísica Óptica y Electrónica (INAOE), Luis Enrique Erro 1, Santa Maria Tonatzintla, 72840 Puebla, Mexico

## Abstract

Falls are a multifactorial cause of injuries for older people. Subjects with osteoporosis are particularly vulnerable to falls. We study the performance of different computational methods to identify people with osteoporosis who experience a fall by analysing balance parameters. Balance parameters, from eyes open and closed posturographic studies, and prospective registration of falls were obtained from a sample of 126 community-dwelling older women with osteoporosis (age 74.3 ± 6.3) using World Health Organization Questionnaire for the study of falls during a follow-up of 2.5 years. We analyzed model performance to determine falls of every developed model and to validate the relevance of the selected parameter sets. The principal findings of this research were (1) models built using oversampling methods with either IBk (KNN) or Random Forest classifier can be considered good options for a predictive clinical test and (2) feature selection for minority class (FSMC) method selected previously unnoticed balance parameters, which implies that intelligent computing methods can extract useful information with attributes which otherwise are disregarded by experts. Finally, the results obtained suggest that Random Forest classifier using the oversampling method to balance the data independent of the set of variables used got the best overall performance in measures of sensitivity (>0.71), specificity (>0.18), positive predictive value (PPV >0.74), and negative predictive value (NPV >0.66) independent of the set of variables used. Although the IBk classifier was built with oversampling data considering information from both eyes opened and closed, using all variables got the best performance (sensitivity >0.81, specificity >0.19, PPV = 0.97, and NPV = 0.66).

## 1. Introduction

Falls are a major threat to the quality of life of older adults. The risk of falling is multifactorial but can be decreased if predisposing factors are addressed [1]. Therefore, the identification of predisposing factors is essential. Clinical guidelines recommend screening the risk of falling in older adults at least once a year [1, 2]. Among identified predisposing factors, balance, [3] aging, [4], and osteoporosis [5] have been found to be the most relevant. Several methods have been developed to assess balance problems and the risk of falling in the elderly population with positive results [4, 6]. However, the use of clinical scales may be insufficient to predict falls in special population such as people suffering from osteoporosis [5]. It has been reported that women with osteoporosis present balance particularities which compromise their stability and predispose them to fall [7]. But while some studies have reported differences in balance among older people with osteoporosis who have fallen compared to older people with osteoporosis who have not [8–10], others have reported no differences [11, 12].

As can be seen, there is a lack of information about the usefulness of objective measures such as postural sway parameters to identify fallers in older people with osteoporosis. Therefore, it is of interest to answer the following research question: how to evaluate and to determine the relevance of balance parameters associated with an older adult with osteoporosis being at risk of falling?

Assessment models have been developed to support the identification of useful information for fall prevention. For example, a linear model to predict the risk of falling in older adults based on postural sway parameters presented a better performance (area under the receiver operating characteristic curve (AUC): 0.73; 95% CI: 0.63–0.83) than a model using exclusively clinical parameters (AUC: 0.67; 95% CI: 0.55–0.79) [13]. Other examples are the logistic regression models that were developed to predict the risk of falling in elder people [8–11, 14–16], but the principal limitation of these models is the assumption of linearity between the dependent variable and the independent variables. Other examples are the prediction models based on intelligent computing methods that are thought to be better than regression techniques [17–19]. In the previously cited works, the authors presented results using regression to evaluate the fall risk. However, these studies do not consider balance parameters and lack detailed information regarding the model's performance to determine the risk of fall.

Another computational alternative is machine learning (ML), which is a subset of artificial intelligence which has played a key role in many health-related realms, due to its wide set of techniques, many of which do not assume linearity between the dependent variable and the independent variables like regression models. The application of machine learning techniques in topics related to healthcare has been varied. For example, Srinivas and Salah [20] applied classification techniques, Random Forest, and deep neuronal networks to estimate consultation length and to predict no-shows at a cardiology clinic; in [16], artificial neural networks models and multiple regression models were used to forecast blood supply at blood centers; in [21], supervised machine learning classifiers were induced to develop predictive models that identify the risk of a patient no-show to a clinical site; in [22], the authors compared four ML algorithms, namely, logistic regression, Random Forest, gradient boosting machine, and artificial neural networks to identify which one has the best performance to predict the patient-specific risk of late arrival to some ambulatory care clinics. In general, the research works report an effectiveness of around 80% to predict the event of interest, which provide evidence of the viability to apply ML techniques to help in healthcare problems.

Machine learning techniques have also been used to build models to predict the risk of falling. In [23], the authors developed a dynamic Bayesian network (DBN) from spatiotemporal data for estimating the risk of falling from gait data of women with osteoporosis with a specificity and sensitivity higher than 70.8% and 90.2%, respectively, but they used a small sample size of 18 patients where the number of fallers was greater than the nonfallers. In [24], the authors made a systematic comparison of multifactorial assessment tools and their instrumentation for fall risk classification based on machine learning approaches with a population of 296 community-dwelling older persons, and their best *F*-score measure obtained from several classifiers was 72.85% with Naïve Bayes classifier; they only used spatiotemporal data to build the classifiers. In [25], the authors studied whether deep learning methods using spatiotemporal data can assess fall risk. They used an existing dataset of 296 older adults, and they obtained the best performance of AUC = 0.75. Another example is a convolutional neural network used to predict status about the risk of falling in older adults using data from inertial sensors capture during walking which achieved good results (AUC: 0.75; 95% CI: 0.54–0.92) in the short-term (<6 months), but was not accurate (AUC: 0.56, 95% CI 0.33–0.74) to predict falls in the long term (from 6 to 12 months) [26]. It is important to mention that the results reported in the works cited are a global value, i.e., the authors do not report the score obtained about the faller classification.

In general, previous works cited indicate that impairments of gait and balance are associated with an increased risk of falls. However, there are inconsistencies regarding the characteristics or parameters most predictive of a fall. To advance fall prevention efforts, there is an important need to understand the relationship between balance and fall risk [27], particularly in osteoporotic older people. Another important issue is determining which is the best computational technique or techniques that allow getting a reliable predictive clinical test to identify the risk of fall because previous works report different types of techniques applied to determine that risk.

In this research, we propose using three machine learning methods to identify elder people at risk of fall. Those techniques are (1) feature selection methods, to evaluate and determine the relevance of balance parameters to identify fall risk of the elder people with osteoporosis, (2) classification methods to build a model to predict falls, and (3) sampling techniques to balance data for improving the performance of the classifiers. The latter technique was applied since we worked with unbalanced datasets.

The principal contributions of our research are as follows: (1) we obtained different sets of parameters, and we discussed the consistency of these sets concerning information reported previously and their relevance to identify the risk of fall, (2) we discussed the effectiveness of the different machine learning methods to build a model to predict falls, and we suggest a good combination of balancing data methods with classifier methods to get a reliable predictive clinical test to identify the risk of fall.

## 2. Method

### 2.1. Subjects and Procedures

Community-dwelling women with osteoporosis older than 60 years, able to stand up for 2 min without assistance and to follow instructions, were recruited at the National Institute of Rehabilitation (INR from its acronym in Spanish) in Mexico City. Women were excluded if they had physical or cognitive impairments or any medical condition that could compromise balance function. Bone mineral density (BMD) of all participants was measured using dual-energy X-ray absorptiometry (DXA) scanners (Hologic, Marlborough, MA, USA). Diagnosis of osteoporosis was made based on their DXA results according to World Health Organization (WHO) definitions (T score lower than 2.5 standard deviations of the mean peak bone mass for healthy adults at one or more skeletal sites). Written consent was obtained from all participants, and the study was approved by the Ethical Committee of the Institute. Sociodemographic information including age and comorbidities of volunteers was obtained from patient records and interviews. All subjects underwent quantitative posturography assessment at their enrollment at the INR. Measurements were performed in a reproducible, well-lit environment, with no audio or visual interference.

Static posturography was performed on a force platform (AccuSway, AMTI Inc., Watertown, MA, USA) with a sampling frequency of 120 Hz. Data were acquired using Balance Trainer software (AccuSway, AMTI Inc., Watertown, MA, USA). Center of pressure (COP) coordinates were analyzed in MATLAB (Mathworks, Natick, MA, USA) to calculate displacement, velocity, area, and frequency-related parameters in anterior-posterior, mediolateral, and resultant direction (see Table 1). Force platform was strapped with an antislip plastic cover (0.01 mm thin) with a template of two lines at 30° to standardize individual foot positions for the repeated measurements across participants and during follow-up. Participants stood up on the platform barefooted on a comfortable, double-legged position aligned to the two 30° lines. Outlines of both feet were marked on the plastic cover with a marker. Individual's base of support (BOS) was entered in the Balance Trainer software after the subject leaves the platform.

Thereafter, patients were instructed to stand on the premarked plastic cover with the arms by the sides and eyes open while looking straight ahead.

Women were tested individually within a single session that lasted less than 5 minutes. Static posturography was performed on two 100-second trials at two conditions (eyes open and eyes closed). Between tasks, subjects were allowed to sit down to rest. Only the first 50 seconds of the trial were used for the calculations to avoid boundary effects, and a low pass bidirectional second-order Butterworth filter with a cutoff frequency of 5 Hz was used.

WHO Questionnaire for the study of falls in the elderly (WHO-QSFE) [28] was also applied to each subject at the beginning of the study. Subjects underwent further functional balance and WHO-QSFE assessments every 6 months. For this study, data of 2.5-year follow-up were used due to the increasing loss of participants.

### 2.2. Data Description and Processing

We used balancing data and feature selection techniques with the balance data of the longitudinal study to discover relevant information to determine fall risk.

#### 2.2.1. Balancing Data

A major problem in many domains is that data are often skewed or unbalanced. In our case, we expect the prevalence of falls among the elderly to be low, and this can be mended by sampling the original dataset, either by oversampling the minority class and/or undersampling the majority class [29]. These techniques have proven to be effective and can help to improve the performance of classifiers to identify the class of interest [30–32].

From the study described in Section 2.1, we recorded 527 instances, each one corresponding to 63 balance parameters obtained from the force platform on one patient of the study. We add the fall data of the patient and used it to determine the class of the instance. It is important to comment that we have 401 instances where the patients did not fall (nonfallers), which belong to the majority class, and only 126 instances where the patients fall (fallers), which belong to the minority class. For this reason, we applied two methods to balance the dataset: oversampling (SMOTE) [29] and subsampling with random undersampling (RUS), both of them integrated as part of the Weka software.

#### 2.2.2. Feature Selection

Raw data contain a mixture of attributes, some of which are relevant to making predictions. It is possible to automatically select those features in the data that are most useful or most relevant for a specific problem. This is a process called feature selection, which reduces the attributes' number in the dataset. Few attributes are desirable because they might reduce the model's complexity, and a simpler model is easier to understand and explain. However, the feature selection process imposes an extra effort of trying to get a subset that preserves the performance of the original dataset. In the context of classification, feature selection techniques can be categorized into filter, wrapper, embedded, and hybrid [27].

Five of the feature selection methods were used from Weka [33] corresponding to the most representative of the classification above, and they were ReliefFAtributeEval, OneRAttributeEval, SymetricalUncertAttributeEval, WrapperSubsetEval, CorrelationAttributeEval, and a homemade algorithm called Feature Selection for Minority Class (FSMC) [34].

#### 2.2.3. Construct Validity

Sixty-three balance features from the static posturographic test were obtained. Balance features were included with a reported utility to identify fallers from nonfallers and subjects with osteoporosis from nonosteoporotic subjects. Those features were used to test convergent validity. We also include features previously studied without positive results using logistic regression techniques [8–11, 14, 15], to test discriminant validity.

COP-related features were grouped into four categories: COP displacement, COP displacement speed, based of support, and time of evaluation. The characteristics of displacement and velocity of displacement of the COP have a theoretical relation with the identification of fallers, nonfallers, and subjects with and without osteoporosis. On the other hand, the characteristics related to the base of support and time of evaluation were controlled to have equal or very similar values in all the subjects throughout all the evaluations, so a theoretical relationship with the identification of falls or osteoporosis is not expected.

#### 2.2.4. Weka

Weka is a machine learning software with algorithms for data mining tasks [33]. In our case, we apply different balancing, feature selection, and classification methods to analyze and describe the data.

### 2.3. Machine Learning

In this section, we describe the classification algorithms applied to verify the importance of the information obtained with feature selection techniques to determine fall risk, using the balance parameters. Those algorithms are implemented in various fields such as economy, medicine, finance, and industry [35].

#### 2.3.1. Classification Techniques

Classification is used to determine to which of a set of categories (groups or classes) a new observation or instance belongs, based on a training set of data containing instances whose category or class membership is known. Generally, a classification technique follows three approaches, statistical, machine learning, and neural network [36]. Considering these approaches, we used five of the most common classifiers applied to predict the risk in health-related studies [37], and the description of each classifier can be consulted in [38]. The classifiers used were as follows: Naïve Bayes which is based on the Bayes theorem, LibSVM which builds a hyperplane or set of hyperplanes in a high- or infinite-dimensional space, AdaBoost which is an ensemble method and is made up of multiple classifier algorithms, RandomForest that creates a set of decision trees from a randomly selected subset of the training set, and IBk which implements the *k*-nearest neighbor algorithm.

### 2.4. Experiments

Three datasets (with eyes open, eyes closed, and one merging both datasets) were used. The experiments were divided into three sets of tests. In the first set, we built five models for each of the three datasets using all features and five models corresponding to the five classifiers mentioned in Section 2.3.1, and 10-fold cross-validation was used to evaluate the performance of each model. As a result, we built 15 models for the first experiment set. For the second experiment set, we built five models for each one of three datasets using the parameters selected by FSMC in each one of the datasets, and we applied 10-fold cross-validation to evaluate the models' performance, we also built 15 models for the second experiment set. Finally, in the third experiment set. We built five models for each of three datasets using the merge parameters selected with the five feature selection methods from Weka mentioned in Section 2.2.2, and we applied 10-fold cross-validation to evaluate the models' performance, so we built 15 models for the third experiment set. We repeated the same three sets of tests with the three datasets, balanced using oversampling and using subsampling. In total, we generated 135 models with 45 models for each resampling method that we used.  Figure 1 shows the 45 models built with unbalanced data, and a similar procedure was followed with the data balanced by the two methods used. Specificity and sensitivity, positive predictive value (PPV), and negative predictive value (NPV) were calculated for each model.

## 3. Results

### 3.1. Subject's Characteristics

One hundred and twenty-six subjects were enrolled (mean age 74.3 ± 6.3, height 148.5 ± 6.4, weight 58.3 ± 8.8, BMI 26.5 ± 3.8) by INR, and a static posturography test was performed on a force platform for each one of them. Patients were asked to return every 6 months for new data acquisition (open and close tests), for 2.5 years, between each period. Patients were asked to report by phone call if they suffered a fall, and these data were added to each one of the record (instance) of the patients.

Due to different circumstances, in each new data collection, there was a smaller number of patients; likewise, in each period, a different number of falls was obtained, and these data are shown in Table 2.

Finally, we collected 527 instances for each test (open and close), 401 with falls and 126 without falls. We used all instances to build different classifiers. So, when we applied oversampling methods, we get a dataset with 401 instances with falls and 401 without falls, and when we applied subsampling methods, we get a dataset with 126 instances with falls and 126 without falls.

### 3.2. Set of Balance Parameters to Identify Falls

The variables selection was applied over all the instances.  Figure 2 shows the sets of balance parameters used to build classification models. In both cases, Figure 2 presents the variable selected from the close eyes dataset ( ), open eyes dataset ( ), and merge dataset ( ).

Table 3 presents the number of variables selected in each dataset (close, open, and merge). With each variable selection method, we obtained three different sets, and using each one of the sets, different classifiers were built.

### 3.3. Performance of Computational Models

The results of the models are presented in two parts. First, the effect of balanced and unbalanced datasets was analyzed plotting the performance (true positive rate and false positive rate) for each developed model irrespective of feature selection method or classifier, showing their receiver operating characteristic (ROC) space (see Figure 3(a)). Balancing data using oversampling techniques results in better classification performance. The cluster of oversampling data lies on the upper left quarter of the ROC space (above the reference line) which is desirable for a good classifier. Unbalanced datasets and subsampled datasets result only on a performance near the reference line.

Second, a detailed analysis was performed over feature selection methods, classifiers, and testing conditions which showed a better performance in ROC space (see Figure 3(b)). Specifically, models built with dataset using all parameters and using IBk (KNN) and Random Forest classifiers for open eyes condition (open) and closed eyes condition (close) showed the best performance, sensitivity = 0.81, specificity = 0.19, sensitivity = 0.79, and specificity = 0.21, respectively. Followed by models from datasets using the FMSC feature selection method with closed eyes condition using Random Forest classifier, sensitivity >0.76 and specificity = 0.24. Sensitivity, specificity, positive predictive value (PPV), and negative predictive value (NPV) are presented in Table 4.

### 3.4. Construct Validity

The set of features selected by the FMSC method contains features of the COP displacement and COP displacement speed in the three measurement conditions analyzed (open eyes, closed eyes, and both). Additionally, Weka's methods were picked up by six bases of support features and one duration time feature during all testing conditions: open eyes and closed eyes. They are *x*-coordinates and *y*-coordinates of the base of support position which are not correlated to falls. These features represented from 5% to 20% of the dataset of selected features by the Weka method. In contrast, the FMSC method selected features mostly at closed eyes. It has been thought that balance tests at closed eyes yield more significant results about the assessment of postural balance [3, 39–41]. This deteriorates confidence in the construct validity of the results obtained based on the set of features selected by Weka's methods.

## 4. Discussion

We tested a set of 63 balance parameters to build models to identify fallers among elderly women with osteoporosis. This approach besides being computationally expensive also lacks construct validity due to the fact it includes sources of pure random information which are not logically correlated with the risk of falling such as *x*-*y* coordinates of the base of support. Variable selection is less computationally expensive. Table 3 shows a resume about the number of variables selected by the methods which get an average reduction of 70% in each study condition.

Notably, the FMSC method selected parameters that have been regarded as highly reliable such as the area of sway (Area Efft) [42, 43] and maximum COP displacement in anteroposterior and mediolateral directions (X max, Y max) [42]. On the other hand, some of the selected parameters have been rejected as representatives of postural balance variability by logistic regression techniques such as displacement in the mediolateral, anteroposterior, and resultant direction as well as the area of 95% ellipsoid (X SD, Y SD, unit path, area95) [9, 42]. Some selected parameters by the FMSC method related to displacement in resultant direction (Rdl D avg, Rdl D SD, Path lgth) have not shown properties to distinguish balance peculiarities in either osteoporotic people [8, 39, 44] people or fallers [39, 40, 42].

FMSC method selected some balance parameters with no reports about reliability or utility such as displacement and velocity in both anteroposterior and mediolateral direction, sway area, and Romberg coefficient (X min, X D avg, Y min, area circ, area rect, Vx max, Vx min, Majr95, Minr95, sway range X, path length X, sway ratio Y, RMSVAP, and Romberg). Consequently, it seems that computing methods such as the FMSC method can extract useful information to identify fallers using specific balance parameters which otherwise are disregarded using only logistic regression techniques.

The results presented in Table 4 show that the use of the variables selected by FSMC and Weka's methods, in general, enables building better classifiers for all datasets that were balanced. In this way, we present evidence of the importance of using balanced information to build classifiers.

Regarding the performance of classifiers, as can be seen in Figure 2(a), the classifiers built with balanced datasets using oversampling methods scored better in sensitivity and specificity measures than all the classifiers. A special case of the model is that based on the dataset using all parameters and the IBk classifier (KNN) for open eyes and closed eyes condition (Merged) because our experiments obtained the best result. But, in general, the results show that the classifier which gets better results using each of the variable sets is Random Forest. The results obtained with classifiers built using variables selected with FSMC and Weka's methods were closed to the best score with a reduced number of parameters. Additionally, features selected with FSMC are more significant and in accordance with the literature that reports the use of the balance data to identify fall risk.

We consider that the combination of oversampling and FSMC selection methods using Random Forest classifier is the best option because it leads to classifiers with better performance to identify the risk of falling using potentially valid and relevant information of key features which could be used as markers to distinguish populations.

The performance of developed models is like those reported in the literature. For instance, the model developed by König [14] based on linear regression techniques showed a sensitivity and specificity of 74% and 76% to classify fallers and nonfallers. Other developed models could explain up to 20% of the variance related to falls [9]. The authors in [45] reported a model based on intelligent computing methods using SVMs with an accuracy of 95% with only two features. However, the last model was used only for classifying people with balancing problems and not to identify the risk of falls.

The difference in results could be mainly attributable to the sample conformation, specifically to the proportion of fallers. König studied a population of 42 fallers and 48 nonfallers. Also, the authors [45] trained a classifier with statistical features taken from gait data of 10 elderly healthy people and 10 elderly people with balance problems. In contrast, in our study, we have 401 records without falls and 126 with falls. Therefore, we consider that the results of specificity and sensitivity are more reliable. An abstract of the performance of each one of the classifiers is summarized in Table 4.

### 4.1. Clinical Implications

Because no testing condition (eyes open vs eyes closed) showed a clear advantage, a clinical test should be conducted for both conditions. All those models were built based on balance parameters feasible to be measured in clinical practice using relatively simple equipment such as balance platforms or accelerometers. It is important due to the seriousness of the associated conditions and because it allows the establishment of an intervention to modify the associated risk within a reasonable time frame.

A bigger proportion of fallers within the sample would be desirable for training and tuning the classifiers. In this study, only balance-related parameters were analyzed. However, falls are multifactorial. Therefore, a combination of balance-related parameters with other data such as gait-related parameters could improve the accuracy of results.

## 5. Conclusion

Most of the classifier performance could be considered inferior to practical requirements for a predictive clinical test, except those built using oversampling methods using all features with either IBk or Random Forest classifiers. None of the test condition (eyes closed or eyes open) showed a clear superiority to identify the risk of falling in osteoporotic women. Therefore, we recommend the assessment of balance on both conditions.

The results show that applying the oversampling method to balance open and close eyes datasets and using the selected attributes using our algorithm FMSC for feature selection enable us to build more valid and feasible classifiers to identify fallers with osteoporosis.

## Figures and Tables

**Figure 1:** Graphic description of the mode of creation of the 45 models built with unbalanced data. *B* = Naïve Bayes classifier, *S* = support vector machine classifier, *K* = IBk classifier, *A* = AdaBoost classifier, and *R* = Random Forest classifier.

**Figure 2:** Sets of variables selected using different feature selection methods from eyes open (o), eyes closed (c), and merge datasets. (a) Using FSMC method and (b) using Weka's methods.

**Figure 3:** (a) ROC space of models developed by applying different machine learning techniques to unbalanced dataset (unbalanced) and balanced datasets (subsampling and oversampling), over data acquired at all conditions (open eyes, closed eyes, open eyes and closed eyes), all feature selection methods (FMSC and Weka's methods), and all classification methods (AdaBoost, Naïve Bayes, LibSVM, Random Forest, and IBk). Models of balanced datasets using oversampling techniques have a better performance. (b) ROC space of models developed with balanced data (oversampling) over data acquired at all conditions, using all feature selection methods and all classification methods. The names of each model graphed follow this nomenclature: the first uppercase letter corresponds to set of variables used, *A* = all variables, *F* = variables selected with FSMC, and *W* = variables selected with Weka's methods; the second uppercase letter corresponds to condition, Op = open eyes, Cl = closed eyes, and Me = open eyes and closed eyes; the third uppercase letter corresponds to the dataset used, *O* = oversampling data, and finally the rest of the name correspond to the name of the classifier used. So, A_Me_O_KNN refers to an IBk classifier built with oversampling data with the merged condition using all variables.

**Table 1:** Analyzed balance parameters.

Parameter number	Parameter name	Parameter abbreviation
	Displacement	
	Mediolateral displacement (*X*)	
1	Average	X Avg
2	Maximum	X Max
3	Minimum	X Min
4	Standard Deviation	X SD
5	Skewness	X Skew
6	Kurtosis	X Krts
7	D average	X D Avg
28	Deviation of CoG	DCG X
36	Sway Range	Sway Range X
37	Path length	Path Length X
39	Sway ratio	Sway Ratio X
59	Frequency	X Freq Avg
	Anteroposterior displacement (*Y*)	
8	Average	Y Avg
9	Maximum	Y Max
10	Minimum	Y Min
11	Standard Deviation	Y SD
12	Skewness	Y Skew
13	Kurtosis	Y Krts
14	D average	Y D Avg
29	Deviation of CoG	DCG Y
38	Sway Ratio	Sway Ratio Y
60	Frequency	Y Freq Avg
	Resultant displacement (D)	
15	Radial *D* Average	Rdl D Avg
16	Radial *D* standard deviation	Rdl D SD
20	Path Length	Path Lgth
61	Frequency	Freq Avg
	Area	
17	Circular	Area Circ
18	Rectangular	Area Rect
19	Effective	Area Efft
	Area 95% Ellipsoid	
31	Area	Area95
32	mayor axis	Majr95
33	minor axis	Min95
34	Mayor axis Tangent	Tan95
35	Mayor axis Slope	Slope95
62	Romberg Coefficient	Romberg Coef
22	Path/Area	Path/Area
30	Area Covariance	Cov
	Velocity	
	Mediolateral velocity (*V*_*x*_)	
57	Average	Vx Avg
23	Maximum	Vx Max
24	Minimum	Vx Min
	Anteroposterior velocity (*V*_*y*_)	
58	Average	Vy Avg
25	Maximum	Vy Max
26	Minimum	Vy Min
40	RMS	RMSVAP
	Resultant velocity (*V*)	
21	Unitarian Path Length	Unit Path
27	Average	V Avg
	Base of support (BoS)	
41	X1 coordinate	BoS(0).x
42	Y1 coordinate	BoS(0).y
43	X2 coordinate	BoS(1).x
44	Y2 coordinate	BoS(1).y
45	X3 coordinate	BoS(2).x
46	Y3 coordinate	BoS(2).y
47	X4 coordinate	BoS(3).x
48	Y4 coordinate	BoS(3).y
49	X5 coordinate	BoS(4).x
50	Y5 coordinate	BoS(4).y
51	X6 coordinate	BoS(5).x
52	Y6 coordinate	BoS(5).y
53	X7 coordinate	BoS(6).x
54	Y7 coordinate	BoS(6).y
55	X8 coordinate	BoS(7).x
56	Y8 coordinate	BoS(7).y
63	Time	Time

The table shows the identification number, name, and abbreviation. Parameters are clustered on categories such as displacement on mediolateral direction, displacement on anteroposterior direction, displacement on resultant direction, area, 95% ellipsoid, Romberg coefficient, path/area, covariance, velocity on mediolateral direction, velocity on anteroposterior direction, velocity on resultant direction, the base of support, and time.

**Table 2:** Instances relation during the study time.

		Follow-up (months)				
Instances	Baseline	First (6)	Second (12)	Third (18)	Fourth (24)	Fifth (30)
Total	126	115	96	81	68	41
Fallers	43	29	27	16	10	1
Nonfallers	83	86	69	65	58	40

**Table 3:** The number of variables selected from each dataset by the selection methods used.

FSMC method				Weka's methods		
Variables	Close	Open	Merge	Close	Open	Merge
Total	63	63	126	63	63	126
Selected	25	13	34	19	10	40

**Table 4:** Specificity (S), sensitivity (Se), positive predictive value (P), and negative predictive value (N) measures obtained with the different classifiers using FSMC's variables (FSMC), Weka's variables (Weka), and all variables (all). AdaBoost (meta), Naïve Bayes (Bayes), IBk (KNN), LibSVM (SVM), and Random Forest (tree) classifiers were built using balanced datasets with the oversampling method. Measures in bold = best classifiers' performance.

			Open eyes					Closed eyes					Merge				
			Meta	Bayes	KNN	SVM	Tree	Meta	Bayes	KNN	SVM	Tree	Meta	Bayes	KNN	SVM	Tree
Oversampling data	All	P	0.70	0.78	0.86	0.50	**0.82**	0.73	0.35	0.91	0.48	**0.85**	0.68	0.71	**0.97**	0.34	0.87
		N	0.53	0.38	0.65	0.96	**0.72**	0.42	0.72	0.65	0.96	**0.73**	0.48	0.56	**0.66**	0.99	0.77
		S	0.39	0.42	0.24	0.27	**0.23**	0.42	0.46	0.22	0.28	**0.21**	0.42	0.37	**0.19**	0.34	0.18
		Se	0.61	0.58	0.76	0.73	**0.77**	0.58	0.54	0.78	0.72	**0.79**	0.58	0.63	**0.81**	0.66	0.82
	FSMC	P	0.62	0.32	0.79	0.60	**0.74**	0.67	0.29	0.84	0.46	**0.83**	0.71	0.31	0.76	0.57	**0.83**
		N	0.52	0.78	0.63	0.60	**0.68**	0.56	0.75	0.67	0.88	**0.70**	0.51	0.76	0.63	0.82	**0.66**
		S	0.43	0.45	0.29	0.40	**0.29**	0.38	0.48	0.25	0.33	**0.24**	0.39	0.47	0.31	0.31	**0.26**
		Se	0.57	0.55	0.71	0.60	**0.71**	0.62	0.52	0.75	0.67	**0.76**	0.61	0.53	0.69	0.69	**0.74**
	Weka	P	0.69	0.69	0.86	0.69	**0.80**	0.66	0.25	0.89	0.79	**0.80**	0.75	0.37	0.87	0.51	**0.81**
		N	0.48	0.44	0.58	0.81	**0.71**	0.46	0.80	0.62	0.65	**0.69**	0.50	0.73	0.63	0.92	**0.73**
		S	0.42	0.44	0.28	0.25	**0.25**	0.44	0.48	0.24	0.28	**0.25**	0.38	0.45	0.25	0.29	**0.23**
		Se	0.59	0.56	0.72	0.75	**0.76**	0.56	0.52	0.76	0.72	**0.75**	0.63	0.55	0.75	0.71	**0.77**

## Data Availability

The data can be provided upon request via email to the corresponding author.
